This article has been retracted.

# Molecular Phylogeny and Revision of Copepod Orders (Crustacea: Copepoda)

**DOI:** 10.1038/s41598-017-06656-4

**Published:** 2017-08-22

**Authors:** Sahar Khodami, J. Vaun McArthur, Leocadio Blanco-Bercial, Pedro Martinez Arbizu

**Affiliations:** 1 Senckenberg am Meer, German Center for Marine Biodiversity Research, Südstrand 44, 26382 Wilhelmshaven, Germany; 2 Savannah River Ecology Laboratory, Aiken, SC USA; 3 Bermuda Institute of Ocean Sciences (BIOS), Hamilton St. Georges, Bermuda

## Abstract

For the first time, the phylogenetic relationships between representatives of all 10 copepod orders have been investigated using 28S and 18S rRNA, Histone H3 protein and COI mtDNA. The monophyly of Copepoda (including Platycopioida Fosshagen, 1985) is demonstrated for the first time using molecular data. Maxillopoda is rejected, as it is a polyphyletic group. The monophyly of the major subgroups of Copepoda, including Progymnoplea Lang, 1948 (=Platycopioida); Neocopepoda Huys and Boxshall, 1991; Gymnoplea Giesbrecht, 1892 (=Calanoida Sars, 1903); and Podoplea Giesbrecht, 1892, are supported in this study. Seven copepod orders are monophyletic, including Platycopioida, Calanoida, Misophrioida Gurney, 1933; Monstrilloida Sars, 1901; Siphonostomatoida Burmeister, 1834; Gelyelloida Huys, 1988; and Mormonilloida Boxshall, 1979. Misophrioida (=Propodoplea Lang, 1948) is the most basal Podoplean order. The order Cyclopoida Burmeister, 1835, is paraphyletic and now encompasses Poecilostomatoida Thorell, 1859, as a sister to the family Schminkepinellidae Martinez Arbizu, 2006. Within Harpacticoida Sars, 1903, both sections, Polyarthra Lang, 1948, and Oligoarthra Lang, 1948, are monophyletic, but not sister groups. The order Canuelloida is proposed while maintaining the order Harpacticoida *s. str*. (Oligoarthra). Cyclopoida, Harpacticoida and Cyclopinidae are redefined, while Canuelloida *ordo. nov*., Smirnovipinidae *fam. nov*. and Cyclopicinidae *fam. nov* are proposed as new taxa.

## Introduction

Copepods are one of the most abundant metazoans on Earth^1^. During their diversification, these small aquatic crustaceans have colonized almost all benthic and planktonic aquatic ecosystems, from deep-sea oceans^2^ to the crevices of the Himalayan glaciers^3^. Copepods are also common parasites of fish and other vertebrates, and many evolutionary lineages live in different degrees of association with invertebrates such as sponges, echinoderms or mollusks^4, 5^.

Despite their important contribution to extant metazoan diversity, especially in the oceans, their phylogenetic position within Arthropoda and the relationships of the major evolutionary lineages within Copepoda (orders in the classification) are still matters of debate. Molecular studies on Copepoda have focused on species- to superfamily-level relationships of Calanoida [e.g., refs 6–10], Harpacticoida (e.g., genus *Tigriopus* Norman, 1868^11^, or Ameiridae^12, 13^), Cyclopoida and Poecilostomatoida (e.g., the families Xarifiidae, Chondracanthidae and Umazuracolidae^14, 15^, Oithonidae^16^ and Cyclopidae^17^).

No molecular ordinal level phylogeny of copepods is currently available, but phylogenetic relationships based on morphological characteristics have been postulated in the past (for a review, see ref. 5). Apomorphies used in morphological analyses are largely based on adaptations (modifications or simplifications) of the locomotory and feeding appendages and body shape to newly colonized environments (e.g., the pelagic realm, crevices of sandy substrates, ground water), and association with invertebrates and fish (including ecto- and endoparasites). In the past, the form of the mouthparts has been considered to be a key evolutionary characteristic complex for the high-level classification of copepods^18^, but this view was not adopted by subsequent authors [e.g., refs 19 and 20]. A comprehensive investigation of homologies in the body plan, segmentation and setation of copepod appendages was performed by Huys and Boxshall^5^, resulting in a cladistics phylogeny of the 10 copepod orders recognized at that time. This concept divides Copepoda into the following three infraclasses: Progymnoplea Lang, 1948 (=Platycopioida Fosshagen, 1985); Gymnoplea Giesbrecht, 1892 (=Calanoida Sars, 1903); and Podoplea Giesbrecht, 1892. The latter was divided into two main clades, the so-called “MHPSM-clade” containing Mormonilloida Boxshall, 1979; Harpacticoida Sars, 1903; Poecilostomatoida Thorell, 1859; Siphonostomatoida Burmeister, 1834; Monstrilloida Sars, 1901; and the “MCG-clade” including the Misophrioida Gurney, 1933; Cyclopoida Burmeister, 1835; and Gelyelloida Huys, 1988. This phylogenetic concept has been revised by many authors^21–26^.

The most important changes to Huys and Boxshall’s^5^ phylogeny were proposed by three authors. a) Martinez Arbizu^21^ first revealed the paraphyletic status of Cyclopoida and Cyclopinidae Sars, 1913. He rejected the ordinal status of Poecilostomatoida and included all of its families in Cyclopoida. b) Dahms^24^ considered the Polyarthra Lang, 1948, to be a separate order of copepods with an uncertain phylogenetic position. c) Ho *et al*.^23^ proposed an ordinal level for the family Thaumatopsyllidae Sars, 1913. These proposals were based on morphological characteristics alone.

Molecular trees resulting from partial taxon sampling incidentally revealed some incongruence with Huys and Boxshall^5^. For instance, Huys *et al*.^14^ considered Harpacticoida to be a sister to Siphonostomatoida, Kim and Kim^27^ and Song *et al*.^28^ questioned the validity of Poecilostomatoida, and Huys *et al*.^29^ considered the Monstrilloida to be a derived clade within Siphonostomatoida.

Discrepancies between trees derived from morphological and molecular data may be due to incomplete taxon sampling, as none of the analyses mentioned above included all 10 orders. Because of the lack of genetic information for many clades of Copepoda, we initiated a comprehensive sampling program to fill the gaps with DNA-suitable material from representatives of all 10 known copepod orders (except the family Thaumatopsyllidae). This dataset includes, for the first time, representatives of the orders Platycopioida, Mormonilloida and Gelyelloida and greatly increased taxon sampling of Harpacticoida and Cyclopoida (including some phylogenetically relevant deep-sea taxa).

The present contribution aims to answer the following three main questions.

1. Is Copepoda (including Platycopioida) a monophyletic group within Pancrustacea? To answer this question, the position of Copepoda was interrogated using 18S rRNA gene sequences of 305 Arthropoda species available from NCBI in addition to our own data from 205 copepod species; together these data include Chelicerata, Myriapoda, Hexapoda, Pentastomida, Ostracoda, Branchiura, Branchiopoda, Remipedia, Cephalocarida, Copepoda, Malacostraca, Thecostraca and Tantulocarida.
2. What are the main evolutionary lineages within Copepoda, i.e., are the subgroups Progymnoplea, Neocopepoda Huys and Boxshall, 1991, and Gymnoplea and Podoplea monophyletic clades?
3. Are the proposed orders of Copepoda monophyletic?

To answer the last two questions, we analyzed 205 species belonging to the orders Calanoida, Cyclopoida, Harpacticoida, Misophrioida, Monstrilloida, Mormonilloida, Platycopioida, Poecilostomatoida, Siphonostomatoida and Gelyelloida using the sequences of genes for the nuclear large (28S) and small (18S) rRNA subunits, cytochrome *c* oxidase subunit I (COI) and Histone 3 protein (H3). Our selection of genes was based on numerous studies using nuclear and/or mitochondrial genes that have resolved phylogenetic relationships between diverse groups [e.g., refs 6, 7 and 30–32].

## Materials and Methods

### Taxon Sampling

The copepod species used in this study were collected from various regions of the world’s oceans, fresh waters and anchialine caves, including the Atlantic and Pacific Oceans, Mediterranean Sea, North Sea, Savannah River (Atlanta, GA, USA) and anchialine caves in Bermuda. Bulk samples were preserved in either 96% ethanol or DESS^33^. More information about sampling sites and collection of the phylogenetically important and rare species representing Platycopioida, Misophrioida, Mormonilloida and Gelyelloida is provided in Supplementary information S1.

Copepod specimens were sorted using a dissecting microscope. Selected specimens were isolated in 96% ethanol or DESS and stored, respectively, at −20 °C or room temperature as vouchers for future reference. Species were selected to represent as many copepod orders and families as possible and were identified to the lowest taxonomic level using diagnostic morphological characteristics. Many of the collected species were new, and, therefore, no specific names can be provided. Collected taxa, sampling coordinates and sequence accession numbers are specified in Supplementary Table S2. We included sequences from GenBank, which added to a total of 205 copepod species representing Platycopioida (2 species), Calanoida (34 species), Misophrioida (8 species), Cyclopoida (28 species), Poecilostomatoida (36 species), Harpacticoida (56 species), Monstrilloida (7 species), Mormonilloida (3 species), Siphonostomatoida (27 species) and Gelyelloida (2 species). Supplementary Table S3 provides a list of the GenBank species and sequences used.

Mystacocarida has been proposed as a sister to Copepoda^34^. We include sequences from both extant genera of Mystacocarida, viz *Derocheilocaris* Pennak and Zinn, 1943, and *Ctenocheilocaris* Renaud-Mornant, 1976 (collected in São Sebastião, São Paulo, Brazil), to test this hypothesis.

### DNA Extraction and Molecular Analyses

DNA extraction from whole individuals were performed using 25–35 μL Chelex (InstaGene Matrix, Bio−Rad) according to the protocol of Estoup *et al*.^35^. From each DNA extract, 20–30 μL of the supernatant was separated from copepod’s voucher specimen, placed in a labeled sterile tube and stored at −20 °C for later DNA analysis. The remaining (generally intact) exoskeletons of the extracted individuals were transferred to glycerin on a glass slide and stored as a voucher for morphological identifications. Genes encoding the nuclear large (28S) and small (18S) subunits of rRNA, Histone 3 protein (H3) and mitochondrial protein cytochrome *c* oxidase subunit I (COI) were used for phylogenetic analysis. Amplification was performed using Illustra PuReTaq Ready−To−Go PCR Beads (GE Healthcare) or AccuStart PCR SuperMix (ThermoFisher Scientific) in a 25-μL volume containing 22 μL H2O or PCR SuperMix, 0.5 μL of each primer (10 pmol μL^−1^) and 2 μL of DNA template. PCR and sequencing primers used for each gene, the length of the amplified regions and the annealing temperature are specified in Supplementary Table S4. PCR products were checked by electrophoresis on a 1% agarose/TAE gel containing 1x GelRed. Forward and reverse sequences for each individual and gene were assembled and edited using Geneious (version 9.1.5 and 5.4.5 Biomatters; http://www.geneious.com). All sequences were searched against the GenBank nucleotide database using BLASTN^36^. Edited DNA sequences for four genes were separately aligned using MAFFT v7.017 under E-INS-i and G-INS-i algorithms^37^ and concatenated using SequenceMatrix 1.7.8^38^. Alignments were further manually edited; regions with ambiguous alignment and an insertion present in seven parasitic poecilostome species (marked in Supplementary Table S3) were excluded from the matrix.

### Phylogenetic Methods

The phylogenetic position of Copepoda within Pancrustacea (Question 1) was examined using the copepod sequences (see above) and 18S rRNA sequences available from GenBank, comprising two species of Mystacocarida, 23 species of Ostracoda, six species of Branchiura, eight species of Pentastomida, 47 species of Branchiopoda, 127 species of Malacostraca, 83 species of Thecostraca, two species of Tantulocarida, one species of Cephalocarida, two species of Remipedia and four species of Hexapoda. The out-group taxa included three species of Myriapoda and Chelicerata. The computationally expensive Maximum Likelihood and bootstrap searches and Bayesian probabilities involving thousands of replicates and millions of generations per data matrix were performed in parallel using grid computing (Linux cluster with 200 cores and 80 GB RAM) at the Senckenberg Biodiversity and Climate Research Center in Frankfurt.

For the Copepoda phylogeny (Questions 2 and 3), nuclear genes (18S and 28S rRNA) and two protein coding genes (COI and H3) were aligned.

Maximum Likelihood analyses were computed using RAxML Ver. 8^39, 40^ under the GTRGAMMAI model of nucleotide substitution following the number of 4 gamma categories and a complete random starting tree (option -d) for the 10,000 bootstrap replicates^41^. The GTRMIX model was performed to select the maximum Likelihood tree with the possibility of optimizing the individual per-site substitution rates for each specified category^41^.

Bayesian analyses were performed with MrBayes MPI version^42, 43^. The best evolutionary model for each gene was calculated using jModeltest v0.1.1^44^.

For protein coding genes (COI and H3), the nucmodel=codon (model GTR) was used [e.g., refs 13 and 45]. Posterior probabilities were estimated using 20,000,000 generations under four simultaneous Markov Chain Monte Carlo chains. A majority rule consensus tree with mean branch lengths was constructed, ignoring the 25% as ‘burn in’ topologies^43^.

### Data Availability

All sequences provided in this study are available from the GenBank sequence database and are listed in Supplementary Table S2.

The resulting alignment and linked trees for both analyses are provided online in the TreeBASE data sharing center at the following web address: http://purl.org/phylo/treebase/phylows/study/TB2:S20470?x-access-code=b15b3fce8b121a31b1583b6096ee5f43&format=html.

### Equipment and Settings

Figures 1, 2 and 3 were modified and homogenized by fonts and sizes in Adobe Photoshop CS2. Figure 4 has been drawn and flattened in Adobe Illustrator CS2. Figure S1 was created using QGIS v 2.14.3-Essen (QGIS code revision: cf2ebb8) under GNU General Public License available from http://qgis.org/en/site/. QGIS Splash screen map courtesy of Stadt Essen. Gridded bathymetry data layer used for the map is provided by ﻿GEBCO available from http://www.gebco.net/data_and_products/gridded_bathymetry_data/.

**Figure 1:** Phylogenetic relationship of Pancrustacea. Phylogenetic relationship of 510 species of Pancrustacea (collapsed to major taxa level) based on 18S rRNA sequences. Numbers show the posterior probabilities calculated by Bayesian analysis.

**Figure 2:** Order-level phylogram of 10 copepod orders. Phylogenetic relationship of 210 copepod species (collapsed to order level) based on Maximum Likelihood and Bayesian analysis of 18S and 28S rRNA, COI mtDNA and H3 histone protein. Nodal support is indicated by posterior probabilities and bootstrap values. Scale bar, nucleotide changes per site.

**Figure 3:** Family level phylogram of Cyclopoida and poecilostomes. Based on Bayesian and Maximum Likelihood analyses of 18S and 28S rRNA, H3 histone protein and COI mtDNA. Nodal support shows posterior probabilities and bootstrap values.

**Figure 4:** New phylogram of copepod Orders. Copepods redrawn from originals: Platycopioida, Calanoida, Canuelloida and Cyclopoida from Sars^19, 30, 82^; Misophrioida from Martinez Arbizu and Jaume^83^ Harpacticoida from Kihara and Martinez Arbizu^84^, Monstrilloida from^85^, Mormonilloida from Huys *et al*.^86^, Gelyelloida from Rouch and Lescher-Moutoué^73^ and Siphonostomatoida from Boxshall and Huys^87^.

## Results

Phylograms related to Pancrustacea and Copepoda are respectively provided in Supplementary Figures S5 and S6; for better visualization, Figures 1 and 2 show trees collapsed to the group level (Pancrustacea) and order level (Copepoda).

### Phylogenetic Position of Copepoda within Pancrustacea (Question 1)

The 18S rRNA alignment for 510 arthropod species comprised 1897 nucleotide positions (1733 bp to 1995 bp). Figure 1 shows the 18S rRNA tree topology and posterior nodal support from Bayesian analyses of Pancrustacea (see Supplementary Figure S5 for the full tree). Malacostraca + (Thecostraca + Tantulocarida) is the sister-group of Copepoda. The present tree shows that Copepoda is a monophyletic group, with Platycopioida (Progymnoplea) as its most basal clade, followed by Calanoida (Gymnoplea) and Podoplea, both also monophyletic. This phylogeny of Pancrustacea agrees with Regier *et al*.^45^ and does not support the monophyly of Maxillopoda. Supplementary Figure S5 shows the full Pancrustacea tree of 18S rRNA and Fig. 1 provides the same tree collapsed at the group level.

### Phylogenetic Relationships within Copepoda (Questions 2 and 3)

Copepoda and the three traditionally accepted infraclasses^5, 46^ were recovered as monophyletic taxa. Progymnoplea (Platycopioida only) was placed in the most basal position in the tree with the sister-group of Neocopepoda (all other orders together), and Gymnoplea (or the highly supported monophyletic Calanoida) was placed as the sister to monophyletic Podoplea (all other copepod orders, Fig. 2).

Within Podoplea, the monophyletic orders Monstrilloida, Misophrioida, Mormonilloida, Siphonostomatoida and Gelyelloida were recovered with high support values. Therefore, the Monstrilloida is retained here as a valid order, as it is not a derived clade within Siphonostomatoida (Supplementary Figure S6).

The Misophrioida is in a basal position within Podoplea, as the sister of all other taxa combined (Fig. 2). Within Misophrioida, the families Speleophriidae (including *Archimisophria*) and Misophriidae were recovered as monophyletic groups (Supplementary Figure S6).

Harpacticoida is shown to be polyphyletic (Fig. 2). Lang’s (1948) Harpacticoid sections Polyarthra and Oligoarthra were each recovered as monophyletic, but they are not sister-groups (Figs 2, S6). Here, we confirm the status of the order Harpacticoida *s. str*. (Oligoarthra) (without Longipedidae and Canuellidae). Consequently, we recognize the formerly known Harpacticoida Polyarthra as a separate order, referring to it as Canuelloida.

The Podoplean clade (Fig. 2) modifies the current phylogenetic interpretation of copepod relationships. The first branch is Misophrioida, followed by two derived clades. Clade 1 comprises Mormonilloida and a sister-group containing the Monstrilloida and Siphonostomatoida (both monophyletic). Clade 2 contains Canuelloida at the base of the clade, followed by Gelyelloida as sister to Harpacticoida (=Oligoarthra) + Cyclopoida (including poecilostomes) (Figs 2 and 3). The Cyclopoida clade (including poecilostomes) is highly supported (Figs 2 and S6). The sister-group of Poecilostomes is the family Schminkepinellidae (Martinez Arbizu, 2006) (Fig. 3), which also showed high support values.

Huys and Boxshall’s^5^ classification of Podoplea into a “MHPSM-clade” (Mormonilloida, Harpacticoida, Poecilostomatoida, Siphonostomatoida and Monstrilloida) and an “MCG-clade” (Misophrioida, Cyclopoida and Gelyelloida) is not supported by our analysis. A synoptic view of the new phylogenetic relationships within Copepoda and the new classification proposed here are depicted in Figure 4.

## Discussion

### Monophyly of Copepoda and its Position within Pancrustacea (Question 1)

The monophyly of Copepoda (including the Platycopioida) within Pancrustacea is demonstrated for the first time. Previous molecular analyses considered only a few species (mostly podopleans) as representatives of Copepoda. Mallat *et al*.^47^ considered a single taxon, identified no further than “Cyclopidae sp.” (Cyclopoida) as a representative for Copepoda in their Ecdysozoan phylogeny, based on 18S and 28S rRNA genes. Regier *et al*.^45, 48, 49^ explored the phylogenetic relationships of Arthropoda using 41 kb of nuclear protein-coding genes, but included only three copepod species, namely one derived Calanoida and two fresh-water Cyclopoida in the analysis. Von Reumont *et al*.^50^, presented an analysis of Pancrustacea using 454 expressed sequence tags (EST) from 1,886 genes, but included just one Harpacticoida species and four species of Siphonostomatoida in the analysis.

The present 18S rRNA tree (Fig. 1) does not support the traditional morphological hypotheses that place Copepoda as the sister-group to the Mystacocarida, within Maxillopoda [e.g., refs 4 and 34]. We include, for the first time, both extant genera of Mystacocarida (*Derocheilocaris* and *Ctenocheilocaris*) in a molecular tree. The tree shows that 1) Mystacocarida is not a sister to Copepoda but to Ostracoda and 2) Mystacocarida + Ostracoda are not closely related to Copepoda; therefore, Maxillopoda must be rejected as a natural group. Its members are distributed into two non-sister major clades in the tree, with the clade consisting of Mystacocarida + Ostracoda, and Pentastomida + Branchiura placed at the base of the Pancrustacea tree. 3) Copepoda is sister to a clade comprising Thecostraca + Tantulocarida and Malacostraca.

All three conclusions have been partially revealed in previous molecular reconstructions of arthropod or pancrustacean phylogenies^45, 51, 52^, but the consequences have never been discussed in detail. It is remarkable that our tree, based on a partial 18S rRNA gene alone (1.7 kb), shows almost the same topology as that of Regier *et al*.^48^, which is based on 62 nuclear protein coding genes (41 kb), although Regier *et al*.^48^. obtained better support values. Regarding Pancrustacea, both analyses differ only in that Regier’s *et al*.^48^ tree does not include Tantulocarida, and Mystacocarida is sister to Ostracoda in the present study but is the sister-group of Pentastomida + Branchiura in Regier *et al*.^48^. Pancrustacea (Hexapoda plus Crustacea) hypothesis is supported here, and, for the first time, the position of Tantulocarida is demonstrated to be a sister-group (outside not inside) to Thecostraca (as compared to the discussion of Petrunina *et al*.^52^).

The lack of support for Maxillopoda as a monophyletic group will have implications for the study of arthropod limb evolution and the re-interpretation of Cambrian Orsten-type fossils^53–55^. Our pancrustacean tree could explain why copepods have never been found in the Orsten fauna; meanwhile, other “maxillopodans” (e.g., Pentastomida) have been reported from these Lagerstätten. The Copepoda + Thecostraca + Tantulocarida + Malacostraca clade (Multicrustacea) must have evolved later in earth history from a Cambrian stem group. The position of the Orsten fossil *Bredocaris* Muller, 1983, close to Thecostraca, is unclear^56^. Additionally, to our knowledge, no Cambrian fossil unequivocally assigned to Thecostraca or Malacostraca. The oldest fossil copepod remains are some legs preserved in 303 Ma old Carboniferous bitumen from Oman^55^. For a review and discussion of fossils assigned to Copepoda, see Selden *et al*.^58^.

The evolution of Copepoda as a progenetic malacostracan was proposed by Gurney^59^ who compared the morphology of the larval “copepodid” stages of copepods to the protozoea of peneid shrimps. This hypothesis was elaborated further by Newman^60^, who extended this idea to the origin of Maxillopoda from Eumalacostraca through progenesis. However, the arguments to support a maxillopodan-malacostracan relationship (or common origin) were mostly based on detailed morphological and developmental patterns of Copepoda and Thecostraca alone^61^, leaving other maxillopodans aside because of a lack of detailed information. Although our Pancrustacea tree invalidates the progenetic origin of Maxillopoda from an eumalacostracan, the progenetic origin of Copepoda from a stem line group common to Communostraca remains a valid hypothesis. Copepoda have developed a terminal moult (adult copepods do not moult further), suppressing the part of development that would be homologous to postlarval development in decapods.

The present phylogeny also resolves the incorrect assumption that Mystacocarida represents the sister-group to Copepoda. This assumption guided Ferrari *et al*.^61^ to an unsupportable interpretation of the evolution of the body plan within Copepoda, inverting the polarity of the transformation series when they proposed the gymnoplean tagmosis as the most derived condition (see below).

The monophyly of Copepoda, as presented here, allows the confirmation of some synapomorphies for the group, for example, the lack of compound eyes during any developmental stage (including the adult stage). The lack of compound eyes prevents the inclusion of the 477–485 Ma Orsten-type fossils with stalked complex eyes, and claims copepod affinities^62^ within Copepoda. Additionally, the suppression of moults in the adult phase can be interpreted as a synapomorphy of Copepoda.

### Major Subdivisions of Copepoda (Question 2)

The phylogenetic relationships within Copepoda, as presented here, reinstate Lang’s major subdivisions^46^. Although not strictly applying the principles of phylogenetic systematics^63^, the argumentation of Lang was always formulated in the context of character evolution. Lang^46^ rejected the major classification of copepods based on mouthpart morphology by Thorell^18^ and claimed that parasitic groups should be classified with the free-living forms ‘they derived from’. He also recognized that in Giesbrecht’s subdivision of the whole Copepoda into 2 single groups, the Gymnopleoden and the Podopleoden groups^20^, which was based on body tagmosis, was insufficient to resolve the basal phylogeny of the group. For the first time, Lang claimed that platycopioids were the most primitive among all copepods and proposed the name Progymnoplea (=Platycopioida) to accommodate them as a first offshoot in the phylogeny of Copepoda, and as a sister-group to all other groups, followed by Gymnoplea (=Calanoida) as the sister-group of a clade comprising Progymnoplea (=Misophrioida) and Podoplea (Harpacticoida and Cyclopoida including poecilostomes and siphonostomes along with free-living forms).

The major articulation between the fifth pedigerous and the genital somites (gymnoplean tagmosis), as presented in both Platycopioida and Calanoida, should therefore be interpreted as a plesiomorphy; therefore, it cannot be used to advocate a Gymnoplean clade comprising Platycopioida and Calanoida, as suggested by Ferrari *et al*.^61^. However, the additional articulation between the fourth and the fifth pedigerous somites (podoplean tagmosis) should be interpreted as a synapomorphy of Podoplea.

The present phylogeny consistently supports the monophyly of the Neocopepoda, Calanoida and Podoplea. Podoplea is a strongly supported monophyletic clade congruent with the strong morphological synapomorphies defined in Martinez Arbizu^21^, including the “podoplean articulation” in body tagmosis, spermatophores stored in the genital somite rather than in the prosome, a maximum of one outer seta on third endopodal segment of legs 2 to 4 and a 1-segmented endopod of leg 5.

### Monophyly and Relationships of Copepod Orders (Question 3)

The Calanoida is the most basal taxon of the Neocopepoda, the sister-group of Podoplea. The four gene analyses recovered a similar topology to the most accepted calanoid phylogeny^10, 64–66^. This analysis recovered all recognized superfamilies within Calanoida and resolved the relationships between Megacalanoidea, Eucalanoidea and Bathypontioidea (including the Fosshageniidae as part of Bathypontioidea)^10^. These relationships should be considered with caution due to the lack of any representative from Ryocalanoidea. Family relationships within the superfamilies were not consistently supported throughout the tree; in any case, the lack of some families and Ryocalanoidea or Epacteriscidae would again make any conclusion less than definitive.

Misophrioida is a strong monophyletic clade placed in a basal position within Podoplea (Fig. 2). This conclusion disagrees with the placement of this order as a sister-group of cyclopoids and gelyelloids by Huys and Boxshall^5^, based on synapomorphies of fused specific antennary exopodal segments and the loss of setae on the exopod of P5. Ho^67^ and later Martinez Arbizu^68^ already argued against the clustering of Misophrioida, together with cyclopoids and gelyelloids, and postulated that misophrioids likely represent a branch that diverged early from the podoplean lineage within Copepoda. Two monophyletic groups within Misophrioida were revealed in the present analysis (Supplementary Figure S6), which agrees with the traditional classification of this order into the *Misophria* group and the *Archimisophria* group^69^. Boxshall and Jaume^69^ raised these groups to the family level (Misophriidae and Speleophriidae, respectively), together with a third monotypic family, Palpophriidae Boxshall and Jaume, 2000, which we were unable to re-collect.

The position of Mormonilloida as a sister-group of Siphonostomatoida + Monstrilloida is strongly supported. There are numerous apomorphies for mormonilloids, most of which are unique to this order (see Huys and Boxshall^5^).

Siphonostomatoida were recovered as a monophyletic group in agreement with the following apomorphies: possession of a one-segmented antennary exopod and a strong modification of labrum and labium into an oral cone that develops into a tapering siphon-like structure in advanced lineages^5, 70^. The monophyletic nature of this group was challenged by Marcotte^71^, who proposed a diphyletic origin for the families associated with fish or other vertebrates from various cyclopoids ancestors. This hypothesis was convincingly rejected by Huys and Boxshall^5^, who considered Siphonostomatoida to be monophyletic. Later, Huys^29^ proposed the inclusion of the Monstrilloida as a derived branch within Siphonostomatoida, arguing in favor of a paraphyletic condition of the later order. He interpreted the structure present on the ventral surface of the cephalothorax in adult monstrilloids to be a reduced siphon. The present results strongly support the monophyly of Siphonostomatoida, placing Monstrilloida as its sister-group (Fig. 2). In the Boxshall scheme^72^ on the phylogeny of copepods, Siphonostomatoida was placed as a sister-group to a clade containing Monstrilloida and Poecilostomatoida + Cyclopoida, based on the synapomorphies’ possession of, at most, a one-segmented antennary exopod, and the loss of the whole exopod in most derived three orders. This assumption was later questioned by Huys and Boxshall^5^ and Martinez Arbizu^21^ due to the lack of whole antenna in monstrilloids, which makes it difficult to confirm whether the exopod was lost.

The monophyly of Harpacticoida is controversial. Huys and Boxshall^5^ hypothesized the following apomorphies for Harpacticoida: fusion of antennulary segments II-VII, IX-XIV, XV-XVII and XVIII-XX in females and III-VIII, IX-XII and XIV-XVI in males, the presence of just three setae on the inner margin of exopodal segment 3 of leg 2, a single seta on inner margin of endopodal segment 2 of leg 1 and a two-segmented maxillipedal endopodite. Dahms^24, 73^ performed the most comprehensive study of postembryonic development of Copepoda and Harpacticoida. He was unable to find any synapomorphy for Harpacticoida *sensu* Lang, although he found that Polyarthra and Oligoarthra were monophyletic. Dahms^24^ was the first to propose the exclusion of the Polyarthra families from Harpacticoida, but did not resolve the position of this taxon within (or outside) Copepoda. Later, Schizas *et al*.^26^ confirmed the exclusion of Polyarthra from Harpacticoida using 28S rRNA. According to Dahms^24^, after the exclusion of Polyarthra, Harpacticoida *s. str*. can be defined by the following four naupliar synapomorphies: the postmaxillary limbs are widely spaced, the antennal coxa^74^ has a strong gnathobase, and the antennal and mandibular endopodites are elongated. The molecular information in our study confirmed the non-monophyletic status of Harpacticoida *sensu* Lang. We propose to follow Dahms^24^ and consider Polyarthra as a separate order, which we formally name Canuelloida. Canuelloida is a well-supported monophyletic lineage within Podoplea.

Gelyellidae were described as a family within Harpacticoida, based on a combination of characteristics from both Polyarthra and Oligoarthra^74^. Later, Huys^75^ excluded Gelyellidae from Harpacticoida, based on a series of mouthpart morphology characteristics, and considered them a separate order with a long evolutionary history that was an early offshoot of the Cyclopoida lineage. Several apomorphies are unique characteristics of this order, including extreme modifications (mostly reductions) to mouth appendages and swimming legs^75^. It is almost impossible to unravel the phylogenetic position of Gelyelloida using morphological characteristics alone. The present molecular tree supports the basal position of Gelyelloida in a clade containing Cyclopoida and Harpacticoida *s. str*. The two new species of Gelyelloida discovered in South Carolina will likely belong to a new genus (J. Reid, com. pers.), but they also present great reductions in segmentation and setation of appendages and will not add much to the discussion at an ordinal level.

The phylogenetic status of Cyclopoida is controversial in the history of copepod classification. Thorell^18^ considered Gnathostoma, Siphonostoma and Poecilostoma to be subgroups of Cyclopoida. Kabata^70^ divided cyclopoids into three separate orders, with poecilostomatoids and siphonostomatoids closer together. Huys and Boxshall^5^ considered Poecilostomatoida and Cyclopoida to belong to separate lineages within Podoplea. This was questioned later by Martinez Arbizu^21^, who indicated that Cyclopinidae Sars, 1913 and Cyclopoida were paraphyletic groups and considered the poecilostomes to be a derived branch of the “Cyclopinidae-lineage” sister to the family Schminkepinellidae. The present molecular results support Martinez Arbizu’s cyclopoid-poecilostome lineage and the derived position of poecilostomes, a sister to the Schminkepinellidae within Cyclopoida. Our phylogeny further confirms the paraphyly of Cyclopinidae (Fig. 3), reinforcing and supporting the split of this family into several monophyletic units of family rank, as proposed by Martinez Arbizu^21, 76–81^. The phylogeny also recovers the gradual invasion of fresh waters by the Cyclopidae Raffinesque, 1815. The most basal group is marine Euryteinae Monchenko, 1974, which is followed by brackish water Halicyclopinae Kiefer, 1927, and finally fresh water Eucyclopinae Kiefer, 1927, and Cyclopinae Dana, 1853. The basal position of *Cyclopicina* Lindberg, 1953, relative to all other cyclopoid families, suggests that this lineage should be raised to the family rank (Cyclopicinidae fam. nov., Supplementary information S7).

### Systematic part

The new phylogenetic relationships within Copepoda proposed here include the definition of new taxa and amendment of some diagnoses. Therefore, redefinition of the copepod orders Cyclopoida and Harpacticoida, definition of order Canuelloida ordo nov., family Cyclopicinidae fam. nov., and Smirnovipinidae fam. nov. are provided in Supplementary information S7.

### Statement of Approval

The copepod species from this study were collected worldwide; a permit was issued to PMA from the U.S. Department of Energy to enter the Savannah River Site. Sampling in Bermuda anchialine caves was made possible by the permission of the Bermuda Department of Conservation Services (contribution, #257), Bermuda Biodiversity Project (BBP), Bermuda Aquarium, Museum and Zoo, Department of Environment & Natural Resources. Marine species were sampled during the IceAGE cruise (Me 85-3), Kurambio-II cruise (SO250, grant 03G0250B), DIVA-III (Me 79-1), EcoResponse (SO239, grant 03F0707E, JPI-Oceans “Ecological Aspects of Deep-Sea Mining” approval and funding from the European Union Seventh Framework Programme FP7/2007–2013) and Abyssline-1 cruise, approved by UK Seabed Resources.

## Electronic supplementary material

Supplementary information online
